This article has been retracted.

# Universal minicircle sequence binding protein of *Leishmania donovani* regulates pathogenicity by controlling expression of cytochrome-b

**DOI:** 10.1186/s13578-016-0072-z

**Published:** 2016-02-17

**Authors:** Ruby Singh, Bidyut Purkait, Kumar Abhishek, Savita Saini, Sushmita Das, Sudha Verma, Abhishek Mandal, Ayan Kr. Ghosh, Yousuf Ansari, Ashish Kumar, Abul H. Sardar, Ajay Kumar, Pradeep Parrack, Pradeep Das

**Affiliations:** Department of Molecular Parasitology and Bioinformatics, Rajendra Memorial Research Institute of Medical Sciences (RMRIMS), Indian Council of Medical Research (ICMR), Agamkuan, Patna, Bihar 800007 India; Department of Biotechnology, National Institute of Pharmaceutical Education and Research (NIPER), Hajipur, Vaishali, Bihar 844101 India; Department of Microbiology, All India Institute of Medical Sciences (AIIMS), Patna, 801105 India; Department of Biochemistry, Bose Institute, Kolkata, 700009 India

**Keywords:** *Leishmania donovani*, kDNA, UMSBP, CBRL, ETC, Apoptosis, Oxidative phosphorylation

## Abstract

**Background:**

*Leishmania* contains a concatenated mitochondrial DNA, kDNA. Universal minicircle sequence binding protein (UMSBP), a mitochondrial protein, initiates kDNA replication by binding with a conserved universal minicircle sequence (UMS) of kDNA. Here, we describe first time in *L. donovani* the regulation of DNA binding activity of UMSBP and the role of UMSBP in virulence.

**Methods:**

Insilco and EMSA study were performed to show UMS-binding activity of UMSBP. Tryparedoxin(TXN)-tryparedoxin peroxidase(TXNPx) assay as well as co-overexpression of cytochrome-b5 reductase-like protein (CBRL) and tryparedoxin in *L. donovani* were done to know the regulation of DNA binding activity of UMSBP. Knockout and episomal-expression constructs of UMSBP were transfected in *L. donovani*. The cell viability assay and immunofluorescence study to know the status of kDNA were performed. Macrophages were infected with transfected parasites. mRNA level of cytochrome b, activity of complex-III, intracellular ATP level of both transfected promastigotes and amastigotes as well as ROS concentration and the level of apoptosis of transfected promastigotes were measured. Level of oxidative phosphorylation of both transfected and un-transfected amastigotes were compared. Burden of transfected amastigotes in both macrophages and BALB/c mice were measured.

**Results:**

*L. donovani* UMSBP is capable of binding with UMS, regulated by redox through mitochondrial enzymes, TXN, TXNPx and CBRL. Depletion of UMSBP (LdU^−/−^) caused kDNA loss, which decreased cytochrome-b expression [component of complex-III of electron transport chain (ETC)] and leads to the disruption of complex-III activity, decreased ATP generation, increased ROS level and promastigotes exhibited apoptosis like death. Interestingly, single knockout of UMSBP (LdU^−/+^) has no effect on promastigotes survival. However, single knockout in intracellular amastigotes demonstrate loss of mRNA level of cytochrome-b, disruption in the activity of complex-III and reduced production of ATP in amastigotes than wild type. This process interfere with the oxidative-phosphorylation and thereby completely inhibit the intracellular proliferation of LdU^−/+^ amastigotes in human macrophages and in BALB/c mice. Amastigotes proliferation was restored as wild type after episomal expression of LdUMSBP in LdU^−/+^ parasites (LdU^−/+^AB).

**Conclusion:**

The LdUMSBP regulates leishmanial mitochondrial respiration and pathogenesis. So, LdUMSBP may be an attractive target for rational drug designing and LdU^−/+^ parasites could be considered as a live attenuated vaccine candidate against visceral leishmaniasis.

**Electronic supplementary material:**

The online version of this article (doi:10.1186/s13578-016-0072-z) contains supplementary material, which is available to authorized users.

## Background

Leishmaniasis presents a spectrum of disease ranging from self-limited cutaneous ulcers to erosive and disfiguring mucocutaneous disease to lethal visceral infections [1]. Visceral leishmaniasis (VL) occurs in 98 countries worldwide however six countries viz., India, Bangladesh, Sudan, South Sudan, Brazil and Ethiopia contributes more than 90 % of global VL cases [2, 3]. VL is caused by the sand fly and transmitted by intracellular protozoan parasite *Leishmania donovani* (belonging to order Kinetoplastida) has been reported in West Bengal, Uttar Pradesh and Bihar in India and poses a worrying health problem in Bihar (accounting for nearly 90 % of the total cases in India) [4]. The defining characteristics of Kinetoplastid order is a highly unusual, concatenated mitochondrial DNA structure, the kDNA (kinetoplast DNA) [5]. kDNA consists of two types of circular DNA viz:, maxicircle [20,000–40,000 base pairs (bp) and present in 10–20 copies] and minicircle (<1000 bp), present in 10,000 copies [6]. Maxicircle contains mitochondrial genes encoding mitochondrial proteins and rRNA. Minicircles encode guide RNAs, function in the process of mRNA editing [7, 8]. One short sequence, universal minicircle sequence (UMS) (GGGGTTGGTGTA), located at the minicircle’s replication origin and is conserved in all trypanosomatid species studied till date [9, 10]. In *Crithidia fasciculata*, UMSBP binds specifically to the UMS and initiates kDNA replication [11, 12] and this UMS-binding activity is sensitive to redox potential [13]. Moreover, at the kDNA replication origin of *Trypanosoma* UMS binding activity of UMSBP is opposingly regulated by mitochondrial redox regulating enzymes, tryparedoxin (TXN) and tryparedoxin peroxidase (TXNPx) [14, 15].

Previous report in *C. fasciculata* suggests the post replication functions of UMSBP [16]. kDNA encodes the mitochondrial genes which participate in electron transport chain (ETC) and leads to ATP generation for proper functioning of parasites [17]. Diskinetoplastidy (loss of kDNA) as well as inhibition of Electron Transport Chain with antimycin A induces apoptotic like death in *L. donovani* parasites [18, 19]. In *Leishmania*, inhibition of ETC complexes reduces amastigotes cell growth. [20]. As UMSBP is involved in kDNA replication, it may also be possible that it involved in parasite survival by controlling the activity of ETC which need further investigation. Moreover, in *T. brucei*, another mitochondrial protein, cytochrome b5 reductase-like protein (CBRL) indirectly regulates the oxidation/reduction status of UMSBP through the oxidation of TXN [21]. However, the regulatory mechanism that mediates oxidation/reduction as well as UMS-binding activity of UMSBP in *L. donovani* remains unknown.

Here, we present the finding on the sequence and structure conservation of LdUMSBP (*Leishmania donovani* UMSBP) and it’s binding with UMS of kDNA. We also demonstrate the redox regulation of UMS-binding activity of LdUMSBP. To know more about UMSBP; biological role other than kDNA replication the UMSBP gene was depleted from promastigote and amastigotes. It was observed that LdUMSBP depletion (LdU^−/−^) induces loss of kDNA and kDNA encoded cytochrome-b (Cyt.b) (essential component of Complex-III of ETC) which induces apoptotic-like phenomena through inactivation of Complex III in promastigotes. Single allele deletion of LdUMSBP (LdU^−/+^) has no role in promastigotes survival. Interestingly, deletion of one allele (LdU^−/+^) is sufficient to completely reduce amastigotes survival. Moreover, in intracellular amastigotes LdUMSBP was found to be necessary for Complex-III activity and LdU^−/+^ parasites shows reduced ATP production by interfering with oxidative phosphorylation than wild type (WT) and are less virulent both in human macrophages and in BALB/c mice. These finding suggests that UMSBP has the role in mitochondrial oxidative phosphorylation necessary for *Leishmania* infection. Such information has potentially useful in determining the physiological functions of LdUMSBP in *Leishmania* cells and help in designing better chemotherapeutic option for VL.

## Methods

### Modelling, interaction and phylogenetic analysis

The sequence of UMSBP (XP_003865287.1) was retrieved from NCBI Protein database [22]. The multiple alignments of LdUMSBP with other group of UMSBPs were analysed in the ClustalW [23]. The model of LdUMSBP was built using Modeller of DSv2.5 [24]. The best model was selected based on DOPE Score [25] and Ramachandran plots [26]. The interaction between the modelled protein and UMS of kDNA was carried out by CDOCKER Program [27] in DSv2.5. The best interacting pose was then selected based on more CDOCKER interaction energy.

### Electrophoretic mobility shift assay (EMSA)

The binding affinity of LdUMSBP with UMS in vitro was analysed by EMSA [28]. Briefly, in 20 μl of standard binding reaction mixture (25 mM Tris–Cl, pH 7.5, 2 mM MgCl_2_, 20 % (vol/vol) glycerol, 1 mg/ml BSA, 25 mg/ml poly(dI-dC)poly(dI-dC) and 12.5 fmol of 5′-^32^P-labeled UMS and 1 mM DTT), purified rLdUMSBP was added and incubated at 30 °C for 30 min and electrophoresed in 8 % native polyacrylamide gel [28] and TAE buffer. Electrophoresis was conducted at 250 V for 1.5 h in 4 °C. Protein–DNA complexes were quantified and analyzed by phosphorimager. One unit of LdUMSBP activity was defined as the amount of protein required for the binding of 1-fmol of the UMS-DNA [11, 12].

### Effect of TXN and TXNPx on LdUMSBP-UMS binding

The effect of TXNPx and TR-TXN-TXNPx-reconstituted reaction on UMS binding of LdUMSBP were analysed as described earlier [16]. The TXN reaction was conducted as described elsewhere [29], with the modifications indicated below. The reaction was conducted under the standard UMSBP-binding assay conditions in the presence of LdUMSBP (0.6 ng) and 12.5 fmol of ^32^P-labeled UMS DNA, as described in EMSA with following modifications: DTT was omitted and the reaction was supplemented with TXN and 20 mM reduced trypanothione [T(SH)_2_]. For the coupling of a T(SH)_2_ reductase, the reaction mixture was supplemented with one unit of trypanothione reductase (TR) per ml and 150 µM NADPH. Reaction was started by the addition of TXN, allowed for 10 min at 30 °C and the products were analyzed by EMSA and quantified by phosphor imaging.

### Generation of overexpressed construct of LdCBRL and LdTXN and transfection in parasites

The LdCBRL and LdTXN ORF were PCR amplified from TOPO-TA-LdCBRL and TOPO-TA-LdTXN construct (generated in our lab) using primers summarised in Table 1. Amplified product of LdCBRL and LdTXN were cloned into *Leishmania* expression-vector, pLGFPN and pLPhyg2 respectively in between the specified restriction sites. The clone pLGFPN-LdCBRL was transfected in parasite by electroporation using a Gene Pulser (Bio-Rad) under conditions described previously [30] to generate CBRL over-expressed (CB+) cell lines and maintained in G418 (50 μg/ml). The CB+ cell lines were co-transfected with pLP-hyg2-LdTXN to generate CB+TXN+ co-transfectant and was maintained in the presence of both G418 (50 μg/ml) and hygromycin B (50 μg/ml). Parasites transfected with the empty vector were used as control.

**Table 1:** Activity of respiratory complex III and of citrate synthase in UMSBP deleted isolated amastigotes for the indicated time point

Specific activity of respiratory complex-III and of citrate synthase in amastigotes isolated from macrophages						
Enzymes	Control (WT)	WT + ANTIMYCINA (72 h)	LdU^−/+^			LdU^−/+^ AB
			24 h	48 h	72 h	72 h
ComplexIII activity/min/mg protein	110.4 ± 9.3	26.4 ± 1.8	45.3 ± 3.2	19.4 ± 1.9	8.2 ± 0.8	104 ± 9.1
Citrate synthase activity	492.5 ± 26.2	–	452 ± 23.1	416 ± 19.8	46 ± 2.8	478.2 ± 24.2

Antimycin A was used as positive control to specifically inhibit complex III. Activity of complex III was reduced significantly compared to the control (WT) in response to LdUMSBP deletion. After episomal expression of WT LdUMSBP in LdU^−/+^ parasites, the activity of complex-III of isolated mitochondria from amastigotes was restored near to WT activity in LdU^−/+^ AB parasites. Citrate synthase was used to monitor the intactness of mitochondria. Up to 48 h of infection, mitochondria was intact and at 72 h mitochondria was disrupted. In add back amastigotes mitochondria were found to be intact

Rates are mean ± SEM

### Oxidation and reduction status of UMSBP by maleimide–polyethylene glycol (PEG)

The oxidation–reduction status of LdUMSBP was monitored by maleimide–polyethylene glycol (PEG) assay [14]. Precisely, lysates prepared from WT, CB+ and CB+TXN+ parasites (500 µg of protein) were treated with 10 mM *N*-ethylmaleimide (Sigma) for 1 h at 0 °C. The *N*-ethylmaleimide was then diluted to 0.1 mM with 20 mM sodium phosphate buffer, pH 7.2, 5 mM EDTA solution and concentrated using a Microcon concentrator (Millipore). Dithiothreitol final concentration 20 mM was added. Lysates were incubated for 1 h at ice followed by extensive dialysis against 20 mM sodium phosphate, pH 7.2 and 5 mM EDTA. The lysates were again concentrated using a Microcon concentrator and 50 µg protein was reacted for 1 h at 0 °C with a 0.3 mM final concentration of PEG (molecular mass of 2385–5000 Da; NEKTAR). The reaction products were analyzed by 5–15 % Tris/glycine SDS-PAGE under reducing conditions and western blot was done using anti-UMSBP antibodies. The bands developed hence analysed through Quantity One software (BioRad).

### Generation of UMSBP knockout parasites

The 0.95 kb flanking sequence upstream (5′F) and 0.90 kb flanking sequence downstream (3′F) of LdUMSBP were PCR amplified using *L. donovani* genomic-DNA using the primers mentioned in Table 1. Both 5′F and 3′F were then cloned in both pX63NEO and pX63HYG vectors in HindIII and SalI as well as SmaI and BglII sites to generate 5′F-pX63HYG-3′F and 5′F-pX63NEO-3′the pXG-PHLEO-LdUMSBP plasmid constructs. Both these circular constructs were then linearized by digestion with HindIII and BglII and two round of transfection was done with these two constructs in *Leishmania*. [30] to generate UMSBP deleted *L. donovani* (LdU^−/−^). Transfectant (LdU^−/−^) resistant to both G418 and hygromycin B were obtained and maintained in RPMI-1640 containing 50 µg/ml G418 and 50 µg/ml hygromycin B.

### Plasmid complementation of LdUMSBP in LdU^−/+^ and LdU^−/−^ parasites

Plasmid complementation experiment was carried out as described earlier [30]. LdU^−/+^ parasite was transfected with the pXG-PHLEO-LdUMSBP plasmid prepared by cloning LdUMSBP ORF in pXG-PHLEO in BamHI site (pXG-PHLEO vector was kind gift from Dr. Stephen M. Beverley, Department of Molecular Microbiology, Washington University in St. Louis) and selected with minimal doses of phleomycin (25 μg/mL) and finally grown in the presence of 50 μg/mL of drug. Also, LdU^−/−^ parasite was transfected with pXG-PHLEO-LdUMSBP plasmid and maintained initially with (25 μg/mL) of phleomycin and finally with 50 μg/mL. The selected cell pools were designated “LdU^−/+^ AB” and “LdU^−/−^ AB” for UMSBP deleted, added back. The presence of episome in AB clones was determined by selectively amplifying LdUMSBP gene using specific pXG-PHLEO backbone primer (5′- CCTCCCCCTGTCCCCGGG-3′) and LdUMSBP reverse one.

### MTT assay to check the cell viability

The MTT assay is a quantitative colorimetric assay for measurement of metabolically active cells. This assay was performed to determine the cell viability of WT, LdU^−/+^, LdU^−/−^, LdU^−/−^AB and AmB treated parasites as described previously [31].

### Semi-quantitative RT-PCR

Reverse transcription was performed as described previously [31]. The synthesized cDNAs were amplified by using PCR primers (Additional file 1: Table S1) for specific genes viz. UMSBP, CBRL, TXN, kDNA, Cyt.b and alpha-tublin (as loading control). The products were run on 2 % agarose gel, stained with ethidium bromide and finally documented and quantified using the Bio-Rad Gel Documentation System and associated Quantity One software.

### DAPI staining for analysis of the kDNA status

DAPI is used for cellular DNA, yielding highly fluorescent nuclei with no detectable cytoplasmic fluorescence [32]. WT, CB+, CB+/TXN+, LdU^−/−^ and LdU^−/−^AB cells were stained with DAPI (50 µg/ml) for 15 min. The stained cells were examined under Fluorescence microscope range 343–445 nm (OLYMPUS).

### Macrophage infection assay

Macrophage infection assay was performed according to the method described earlier [30, 33]. Briefly, 10^4^ THP1 cells (pre-treated with PMA-phorbol myristate acetate) per well on glass cover slips were seeded and allowed to adhere, unattached cells were washed. *Leishmania* promastigotes (WT, LdU^−/+^ and LdU^−/+^AB parasites) were added at a ratio of 1:10 (macrophage: parasite) on adhered macrophages and maintained at 37 °C in 5 % CO_2_ for 6 h. Non-internalised promastigotes were eliminated and the cultures were incubated for 5 days, slides were fixed in absolute methanol, stained with Giemsa stain and the parasite load was determined microscopically.

### Isolation of the intracellular amastigotes from infected macrophages

After 12 h post-infection, human macrophages were suspended in chilled PBS containing 1 mM EDTA and 11 mM Glucose. Then the suspension was passed five times through a 27-gauge needle. Cellular debris was removed by centrifugation (60*g* for 5 min at 4 °C) and the supernatant was passed through a 3 μm pore filter. Intracellular amastigotes were then recovered by centrifugation of the filtrate (800*g* for 10 min) [34].

### Measurement of respiratory complex III and citrate synthase assay

The activity of Complex III was assayed in 50 mM KH_2_PO_4_ buffer (pH 7.4) containing 1 mM EDTA, 50 µM oxidized Cyt.c, 2 mM KCN and 10 µM rotenone. After the addition of ubiquinol 2 (150 µM) the rate of reduction of Cyt.c was measured at 550 nm and antimycin A (400 nm) was added to determine the background rate [35].

Citrate synthase activity was assayed in 100 mM Tris (pH 8.0), 100 µM acetyl CoA, 10 µM DTNB and 50 µg of mitochondrial protein. The reaction was initiated by the addition of 100 µM potassium oxalate and rate of change in absorbance was measured at 412 nm [36].

### Measurement of intracellular ATP

The 1 × 10^6^ promastigotes (WT, LdU^−/+^, LdU^−/−^ and LdU^−/−^AB) were resuspended in reaction buffer containing 1 mM dithiothreitol, 0.5 mM luciferin, and 12.5 µg/ml luciferase and mixed gently, after which readings were taken [37]. ATP standard curve was prepared run in all experiments with different concentrations of ATP, calculations were made against the curve and cellular ATP levels were expressed as nmol/10^6^ cells.

In case of amastigotes, a crude mitochondria preparation from WT, LdU^−/+^ and LdU^−/+^AB amastigotes was obtained as described elsewhere [38]. ATP production was measured in the presence of indicated substrates (succinate, pyruvate and α-ketoglutarate) and 67 μM ADP. Inhibitors (6.7 mM malonate, 33 μg/ml attractyloside) were pre-incubated with mitochondria for 10 min on ice. The concentration of ATP was determined by Luminometer using the ATP Bioluminescence kit CLS II (Roche Applied Science, IN).

### Reactive oxygen species (ROS) measurement

Intracellular levels of ROS of WT, LdU^−/−^, LdU^−/−^AB and antimycin-A treated promastigotes were measured as described earlier [30, 33] using a LS55 spectrofluorimeter (Perkin Elmer) with excitation at 504 nm and emission at 529 nm. AmB treated cells was used as positive control.

### Measurement of mitochondrial membrane potential

Mitochondrial membrane potential (∆Ψ_m_) of WT, LdU^−/−^, LdU^−/−^AB and antimycin-A treated promastigotess was measured using JC-1 probe [20]. Briefly, cells were labeled for 10 min with 10 µM JC-1 at 37 °C, washed, resuspended in PBS. JC-1, a cell-permeable dye exists in a monomeric form that on entering the cytoplasm, emits a green fluorescence and upon entering the mitochondria, it forms aggregates and emits a red fluorescence. The ratio of the reading at 590 nm (red) to the reading at 530 nm (green) (590:530 ratios) was considered as the relative ∆Ψ_m_ value.

### Detection of Cyt c

Release of cytochrome *c* from mitochondria into the cytoplasm of WT, LdU^−/−^, LdU^−/−^AB, antimycin-A treated and AmB treated promastigotes were evaluated by Western immunoblotting using a BD ApoAlert cell fractionation kit following the manufacturer’s instructions (Clontech, Palo Alto, CA, USA) as described by our group [39]. Briefly, cytosolic and mitochondrial fractions were fractionated by differential centrifugation. Proteins samples (50 µg) from cytosolic fractions were separated by 12 % SDS-PAGE and Western immunoblotted with rabbit polyclonal anti-cytochrome c antibody.

### Assessment of apoptosis markers

Annexin-V assay (Phosphatidylserine externalization), DNA fragmentation analysis, metacaspase like protease activity and lactate dehydrogenase assay were carried out in WT, LdU^−/−^, LdU^−/−^AB, Antimycin A treated and AmB treated promastigotes according to our previous work [30]. Detailed methods are given in Additional file 1: Materials and methods.

### Mouse infection

BALB/c mice (n = 3) were infected via tail vein with 3 × 10^6^ metacyclic *L. donovani* promastigotes of either WT or LdU^−/+^ or LdU^−/−^AB parasites. Breifly infective-stage metacyclic promastigotes were isolated from stationary phase cultures by density gradient centrifugation as described [40]. About 6 and 14 weeks post infection, all the mice were sacrificed and parasite burdens of liver and spleen were measured by the serial dilution method [40].

### Ethical statement

For animals use, protocols were reviewed and approved by the Institutional Animal Ethical Committee. The RMRI, ICMR follows ‘‘The Guide for the Care and Use of Laboratory Animals,’’ 8th edition by the Institute for Laboratory Animal Research.

### Statistical analysis

All experiments were conducted at least in triplicate, and the results are expressed as mean ± SEM of three experiments and the data were statistically analyzed by Single ANOVA test. A P value <0.05 was considered significant.

## Results

### UMSBP interacts with UMS of kDNA

In *Trypanosoma*, zinc knuckle of UMSBP was found responsible for DNA binding activity [11, 13, 41]. In *L. donovani* UMSBP, a highly conserved CCHC type zinc knuckle i.e., CX2CX4HX4C (X can be any amino acid) was found (Fig. 1a, b). Two Zinc domain binding sites were also observed in the 3D model of LdUMSBP (DOPE Score −2218.945068 and the number of residues in favored region was 88.5 % in Ramachandran plot) (Additional file 1: Figure S1). The model of LdUMSBP was successfully docked onto the UMS (Fig. 1c). The best protein-DNA interaction has CDOCKER energy and CDOCKER interaction energy was 76.8111 and 738.637 respectively. The interacting residues of LdUMSBP are ARG 83, ARG 91 and CYS 93 (Additional file 1: Table S2).

**Fig. 1:** Computational analysis of LdUMSBP. **a** Multiple Sequence Alignment of LdUMSBP with different UMSBP protein sequences showing the conserved DNA binding domain CX2CX4HX4C. **b** Phylogenetic analysis of LdUMSBP with other UMSBP. **c** Interaction of LdUMSBP with UMS, demonstrated by CDOCKER Program in DSv2.5

In-vitro, the interaction of LdUMSBP with UMS was analysed by EMSA (Fig. 2A). Intensity of UMSBP-UMS complex formation was increased with increasing concentration of UMSBP (Fig. 2A, lanes-b–d) in compare to no protein containing reaction mixture (Fig. 2A, lane-a) where no protein-DNA complex was formed. UMS binding activity (unit) against indicated concentration of rLdUMSBP is graphically represented (Fig. 2B). The EMSA result suggests that rLdUMSBP interacts with UMS of kDNA in vitro.

**Fig. 2:** The binding affinity of purified rLdUMSBP with UMS of kDNA. **A** LdUMSBP of indicated concentrations incubated with 12.5 fmol 5′-P^32^-labeled UMS at 30 °C for 30 min and reaction products were analysed through EMSA showing the band of protein-DNA complex. **B** Graphical representation of quantified data of the EMSA gel. DNA binding activity was expressed in *units*

### TXN and TXNPx oppositely regulate the binding activity of LdUMSBP

We observed that LdUMSBP binds with UMS in its reduced form, not in oxidized form (Additional file 1: Figure S4). In *Crithidia,* TXN reduces the UMSBP and enhances the UMS-binding activity [13]. In our study, the relative UMS-binding activity (%) increases with increasing concentration of TXN (Fig. 3A, Panels A and B, lanes-c, d) in comparison to UMS binding without TXN (Fig. 3A Panel B, lane-b). When the concentration of TXN is kept constant and TXNPx is increased then the relative UMS binding was decreased (Fig. 3B, Panels A and B, lanes-c–e). The above observations clearly suggest that TXN and TXNPx oppositely regulate DNA binding activity of LdUMSBP to UMS.

**Fig. 3:** Reconstituted LdTXN–LdTXNPx reaction regulates the binding of LdUMSBP to UMS DNA. rLdUMSBP was incubated with TXN, as indicated, in a TXN reaction mixture (**A**, *Panel A*) and the reaction was followed by the addition with the indicated concentrations of TXNPx (**B**, *Panel A*) as described under “Methods”, followed by the UMS-binding assay (EMSA). **A**, *Panel B* and **B**, *Panel B* Phosphorimaging quantification of EMSA data. The percentage of complex formation presented relative to the value measured in the absence of TXNPx in a reaction mixture supplemented with 0.9 mM TXN was used as a 100 % (**B** *Panel A*). *Lane-a* of (**A**) and (**B**) correspond to no protein

### CBRL over-expression induces kDNA loss by oxidation-inactivation of LdUMSBP and TXN counter balances the effect of CBRL in vivo

Over-expression of LdCBRL in CB+ (CBRL over-expressing *L. donovani*) cell lines was confirmed by RT-PCR. The band intensity of LdCBRL in CB+ cells was ~3.8-fold higher (p = 0.0055) then the WT parasites (Fig. 4A). The similar observations were also observed in western blot with anti-GFP antibody (Fig. 4B). Moreover, the over-expression of TXN in TXN and CBRL co-overexpressed cells (CB+TXN+) was confirmed by RT-PCR (p = 0.0047) and western blot (p = 0.001) (Fig. 4D, E). Both results clearly suggest that LdCBRL and TXN transcripts are present at high copy numbers in transfectants.

**Fig. 4:** CBRL over-expression induces UMSBP oxidation and kDNA loss whereas TXN co-over-expression in CBRL-OE parasite counter balances the effect of CBRL in vivo. **A**–**F** Confirmation of CBRL and TXN over-expression in CB+ and CB+TXN+. **A**, **D** mRNA level of CBRL and TXN by semiquantitative RT-PCR. *Panel A*—gel images; *Panel B*—densitometry data. **A**–tub (alpha-tubulin) PCR was as loading control. **B** and **E** Western blot analysis of GFP and TXN expression in CB+ and CB+TXN+ parasites respectively and in WT parasite. *Panel A*—gel images; *Panel B*—densitometry data. **C** and **F** The presence of pLGFP-LdCBRL and pLp-NEO2-LdTXN constructs in transfected parasite was detected by PCR. *Lane M*—Marker, *Lane 1* shows the bands obtained by PCR using pLp-NEO2 and GFP vector specific foreward primer (designed from just upstream of the start code of LdTXN and LdCBRL respectively) and LdTXN and LdCBRL specific reverse primer respectively. *Lane 2* shows the band obtained by PCR using gene specific foreward and reverse primers. **G** Oxidation (O-UMSBP) and reduction (R-UMSBP) level of UMSBP in CB+, WT and CB+TXN+ parasites. **H** Level of minicircle DNA (kDNA) in CB+, WT and CB+TXN+ parasites was determined by semi-quantitative RT-PCR. **I** Microscopic analysis by DAPI staining to determine the kDNA loss in WT (**a**), CB+ (**b**) and CB+TXN+ (**c**) parasites. *N* Nucleus, *K* kDNA and *a* loss of kDNA. *Asterisk* denotes that the data are significant (p < 0.01)

In *Trypanosoma* overexpression of LdCBRL leads to oxidation of UMSBP and controls its redox state which induced loss of kDNA [16]. Here, we also observed ~fourfold (p = 0.0015) loss of kDNA in CB+ cells in comparison to WT cells. Moreover, the level of minicircle in WT and CB+ cells using *L. donovani* kDNA specific primers, a ~3.6-fold lower band intensity of minicircle in CB + than in WT cells was observed (Fig. 4H). Thereby suggests that LdCBRL indirectly controls the level of kDNA. We have also demonstrated that redox regulates the binding of LdUMSBP with UMS (Additional file 1: Figure S4) which is responsible for synthesis of kDNA [17]. And possibly that is the reason that oxidation–reduction status of LdUMSBP in CB+ and WT cells were demonstrated in PEG Assay [14] where two bands were noticed on nitrocellulose membrane in CB+ and WT. The intensity of 14 kDa band in WT was more than CB+ and the 20 kDa band intensity in CB+ was 4.1-fold higher than WT cells (Fig. 4G). The 14 and 20 kDa bands represent the reduced and oxidized level of UMSBP respectively. Inversely, TXN co-expression increased the level of reduced LdUMSBP in TXN+CB+ cells by ~2.5-fold than CB+ cells (Fig. 4G). Consequently, a increase level of minicircle was increased in CB+TXN+ cells compared to CB+ cells (Fig. 4H) and gain of kDNA in TXN+CB+ cells was observed (Fig. 4A, B, C). These clearly confirm that LdUMSBP is oxidized in CB+ cells leading to loss of kDNA and TXN counterbalance the effect of CBRL by reducing LdUMSBP.

### Double deletion of LdUMSBP (LdU^−/−^) inhibits minicircle synthesis, induces kDNA loss and reduces cell viability but, single gene deletion (LdU^−/+^) has no effect on promastigotes survival

Double Knockout construct for LdUMSBP gene was generated to demonstrate its function in vivo other than kDNA replication. Two rounds of gene replacement (as the *Leishmania* is asexual diploids) with neomycin and hygromycin selectable markers was carried out (Fig. 5a) [30]. Deletion and replacement of both alleles of LdUMSBP by NEO and HYG genes were confirmed through NEO and HYG gene specific PCR (Additional file 1: Figure S5) as well as through southern blot (Additional file 1: Figure S6) [30]. PCR analysis on genomic DNA with primers generated from the coding region as well as from the 5′- and 3′-flanking regions was done to screen the null mutants (LdU^−/−^) (Fig. 5b). PCR and Western blot were used to confirm the complete loss of UMSBP in LdU^−/−^ and the presence of ~42 % LdUMSBP in the LdU^−/+^ lines (Fig. 5c, d).

**Fig. 5:** Targeted gene replacement of LdUMSBP alleles to make LdUMSBP depleted parasites and its effect on kDNA and parasite survival. **a** Schematic representation of the LdUMSBP locus and the plasmid constructs used for gene replacement. **b** Agarose gel analysis of PCR amplified products of LdUMSBP gene. *Lanes* WT, LdU^−*/*+^ and LdU^−/−^ correspond to PCR with gDNA from WT, LdU^−*/*+^ and LdU^−/−^ parasites respectively with external forward and reverse primers which were generated from 42 base pair upstream of LdUMSBP and position 36 downstream of the stop codon of the gene, respectively. The expected size of LdUMSBP, HYG and NEO PCR products are 1.2, 3.4 and 3.7 kb. **c** The presence of episomal LdUMSBP-pXG-phleo construct in transfected LdU^−/+^ and LdU^−/−^ parasites were detected by the PCR. *Lane 1* and *2* shows the band obtained by PCR using pLp-NEO2 vector specific foreward primer (designed from just upstream of the start code of UMSBP) and LdUMSBP specific reverse primer form LdU^−/+^ and LdU^−/−^ parasites. *Lane* *3* is negative control to show the PCR specificity. *Lane M* is 1 kb marker. Figure shows that the UMSBP deleted parasites contain LdUMSBP ligated in a direct orientation in pXG-phleo vector. **d** Western blot using anti-LdUMSBP antibody to check the level of protein in indicated parasites. *Panel A*—Blot image. *Panel B*—graphical representation of densitometric data **e**–**g** Deletion of LdUMSBP induces kDNA loss and decreases parasite survival. **e** Status of minicircle (kDNA) by semiquantitative RT-PCR of WT, LdU^−*/*+^, LdU^−/−^ and LdU^−/−^AB parasites. *Panel A*—gel image, *Panel B*—graphical representation of the densitometry data. **f** Microscopic analysis of kDNA of WT, LdU^−/−^ and LdU^−/−^AB parasites respectively. **g** Effect of UMSBP knockout on promastigotes survival. Single gene deletion has no effect on parasite survival. AmB was used as positive control. *Asterisk* denotes that the data are significant (p < 0.01)

To analyse the status of kDNA in WT, LdU^−/+^, LdU^−/−^ and LdU^−/−^ AB cells by semi quantitative RT-PCR showed that the band intensity of minicircle in LdU^−/+^ and LdU^−/−^ cells were ~2.5- (p = 0.0021) and ~4.3-fold lower (p = 0.0001) than WT cells (Fig. 5e) and consequently, there was approximately 50 % loss of kDNA in LdU^−/+^ compared to WT. Almost no kDNA was found in LdU^−/−^ cells (Fig. 5f). The cell viability of LdU^−/−^ parasites was also reduced by ~5.0-fold compared to WT parasites, but the cell viability of LdU^−/+^ parasites were similar to WT (Fig. 5g). The change in the level of kDNA minicircle and promastigotes survival was dramatically restored in LdU^−/−^AB parasites (Fig. 5). These results clearly indicate that LdUMSBP is involved in kDNA synthesis is described earlier [17] along with parasite survival.

### Deletion of UMSBP induces apoptotic like phenomena via the disruption of ETC-Complex III and ROS generation

As the Cyt.b is an important component of ETC Complex-III, the mRNA expression of Cyt.b was examined in WT, LdU^−/−^ and LdU^−/−^AB to observe whether the UMSBP deletion causes decrease in Cyt. b or not. mRNA level of Cyt.b was found to be ~fourfold lower (p = 0.00074) in LdU^−/−^ cells compared to WT and the level of Cyt.b was restored as WT in LdU^−/−^AB (Fig. 6a). We then investigated whether decreased expression of Cyt. b could disrupt the activity of Complex III or not. Activity of complex-III was found to be decreased drastically in LdU^−/−^ cells compared to WT (Fig. 6b). Electron transport through complex-III involving Cyt.b is essential for the synthesis of ATP by F1/F0 ATPase (complex-V). A decreased (~fivefold) level of intracellular ATP in LdU^−/−^ parasites (p < 0.0001) compared to WT was observed (Fig. 6c). In LdU^−/−^AB cells the activity of complex-III along with the intracellular level of ATP was restored as in WT (Fig. 6b, c). These results clearly suggest that deletion of LdUMSBP causes depletion of Cyt.b leading to the inactivation of ETC Complex III which reduces the level of intracellular ATP in parasites and thereby reduced parasite survival was observed.

**Fig. 6:** Silencing of LdUMSBP induces Apoptosis like cell death by disrupting the Electron Transport Chain. **a** Expression level of Cyt. b in WT, LdU^−/−^, and LdU^−*/*−^AB parasites by semiquantitative RT-PCR. **b** Specific activity of complex-III of ETC and of citrate synthase activity in WT, LdU^−/−^, and LdU^−/−^AB parasites. **c** Production of intracellular ATP of WT, LdU^−/−^, antimycin A (positive control) treated and LdU^−/−^AB parasites. **d** Oligosomal degradation of DNA of the indicated parasites. Deletion of LdUMSBP induces DNA degradation in LdU^−/−^ parasites. Genetic complementation (LdU^−/−^AB) completely reduces the DNA degradation. **e** Assay of cell death taking the same set of parasite used in DNA degradation assay by flow cytometry. Figure denotes differential changes in apoptotic population (Annexin-V positive but PI negative) (as expressed by % of apoptotic cells) in response to deletion and complementation of LdUMSBP alleles. **f** Graphical representation of % of apoptotic cells. **g** Generation of intracellular ROS by WT, antimycin A treated and LdU^−/−^ parasites. **h** Determination of Ψ_m_ as described in materials and methods of indicated parasites. **i** Western blotting to analyse the release of Cyt. c in the cytosolic fraction in response to deletion of LdUMSBP and Antimycin A treatment. **j** Determination of Metacaspase like protease activity. Increased fluorescence intensity indicates increased metacaspase-like protease activity. **k** Determination of membrane integrity by measuring released lactate dehydrogenase. In all experiments AmB was used as *positive* control. *Asterisk* denotes that the data are significant (p < 0.005)

Inhibition of Complex III induces ROS generation in *L. donovani* [20]. In the present investigation, the level of intracellular ROS was found to be increased ~fourfold in LdU^−/−^ parasites (p < 0.0001) compared to WT (Fig. 6g). Antimycin A treated parasites showed inhibition of complex-III and consequently increased ROS generation (Fig. 6d). The level of intracellular ROS was reduced in LdU^−/−^AB cells as WT (Fig. 6g). Therefore, these findings suggest that deletion of UMSBP increases ROS level in *L. donovani* through the inactivation of Complex III.

It was reported that inhibition of ETC (complex III) induced apoptotic like death via generation of ROS, loss in mitochondrial membrane potential (∆Ψ_m_), release of Cyt.c, DNA fragmentation etc. [20]. Our spectrofluorimetric analysis also showed that deletion of LdUMSBP induced loss in ∆Ψ_m_ ~3.5-fold (p = 0.0024) which is comparable with Antimycin A treated cells (loss in ∆Ψ_m_ ~4-fold, p = 0.0012) (Fig. 6h). And after add back of LdUMSBP, the ∆Ψ_m_ was regained in LdU^−/−^AB parasite (Fig. 6h). Cyt.c, a mitochondrial component of ETC [24] released from mitochondria to cytosol due to loss in ∆Ψ_m_ in LdU^−/−^ cells (Fig. 6i) [24] however, no release of Cyt. c in LdU^−/−^AB was observed (Fig. 6i).

Phosphatidylserine (PS) is externalized on the membrane of apoptotic cells [30, 42]. We observed that UMSBP deletion induced PS externalization on LdU^−/−^ parasites (Fig. 6e) and the % of Annexin-V positive (apoptotic) cells were 44.2 % as compared to WT (~8 %) (p < 0.0001) (Fig. 6f). In case of antimycin-A and AmB,  % of apoptotic cells were 36.2 and 58.6 % respectively which were comparable with UMSBP knockout (44.2 %) (Fig. 6e, f). Whereas,  % of apoptotic cells were decreased significantly in LdU^−/−^AB parasites as in WT compared to LdU^−/−^ parasites (Fig. 6e, f). Therefore, externalization of PS on the membrane of LdU^−/−^ cells induces apoptotic like death by inhibiting ETC. Metacaspase like protease activity was found in apoptotic cells (LdU^−/−^) (Fig. 6j) and interestingly, this activity was reduced significantly in LdU^−/−^AB cells (Fig. 6j) as in WT. Parasites treated with AmB were considered as positive control (Fig. 6j). Lactate dehydrogenase activity assay demonstrated that throughout the apoptotic events, membrane of the LdU^−/−^ parasites were intact (Fig. 6k).

Metazoan apoptosis is characterized by DNA fragmentation [43]. DNA Fragmentation was observed (in multiples of 150 to 200 bp) in LdU^−/−^ cells (Fig. 6d, lane2) which was comparable to DNA fragmentation due to known apoptosis inducer, Antimycin A (Fig. 6d, lane4) and AmB (Fig. 6d, lane5). DNA fragmentation was significantly completely reduced in LdU^−/−^ AB parasites as in WT (Fig. 6d, lane3). Overall, the finding indicates that double deletion of LdUMSBP induced DNA degradation and episomal expression of LdUMSBP in LdU^−/−^ parasites completely abolished the DNA degradation in LdU^−/−^AB cells. Thus, LdUMSBP being a replication initiation enzyme is involved in controlling the apoptosis phenomena in *Leishmania*.

### Deletion of single allele of LdUMSBP (LdU^−/+^) in the intracellular amastigotes reduces ATP production by interfering with oxidative phosphorylation

To confirm the effect of LdUMSBP on ETC-complex-III activity under more physiological conditions, we infected PMA treated THP1 cells with WT, LdU^−/+^ and LdU^−/+^AB promastigotes and from these infected cells, amastigotes were isolated (Fig. 7a). mRNA level of Cyt.b (which is encoded by kDNA and is an indispensible component of complex-III) was found to be significantly lower (p = 0.0018) in the mitochondria of LdU^−/+^ amastigotes compared to the WT (Fig. 7b). This could be probably due to the complex-III activity which was significantly reduced in LdU^−/+^ cells compared to WT (Table 1). Interestingly, the level of Cyt.b and the complex-III activity were regained in LdU^−/+^AB amastigotes (Fig. 7b, Table 1). Also, the citrate synthase activity was reduced significantly in LdU^−/+^ (Table 1), indicating the loss in intactness of mitochondria. We further investigated whether some other component(s) beside Cyt.b are involved in this phenomenon. Since respiratory complex-III is required for ATP production in the mitochondria, we investigated the ATP generation in the indicated parasites after deletion of LdUMSBP. ATP production was highly reduced in LdU^−/+^ parasites (p = 0.0012) compared to the WT parasites (Fig. 7c). In comparison to WT mitochondria ATP generation was reduced to 20 % in LdU^−/+^ amastigotes mitochondria which was further regained in LdU^−/+^AB amastigote (Fig. 7c). LdUMSBP thus found to controls the activity of Complex-III and thereby controls the ATP generation. The involvement of complex-III in ATP production through oxidative phosphorylation was confirmed by measuring its level in presence of substrates that distinguish substrate level phosphorylation from oxidative phosphorylation [44]. The substrate for oxidative phosphorylation is succinate and for substrate level phosphorylation are α-ketoglutarate (of citric acid cycle) and pyruvate. Malonate (inhibitor of succinate dehydrogenase) inhibits the ATP production by oxidative phosphorylation. The attractyloside (inhibitor of mitochondrial import of ADP in the reaction buffer) inhibits the all three forms of ATP production [45]. When the succinate was used as a substrate, the mitochondria of LdU^−/+^ amastigotes produced about 40 % (p = 0.001) of the ATP of WT mitochondria (Fig. 7d). Moreover, LdU^−/+^AB mitochondria restores the ATP production level as in WT whereas, malonate reduces succinate derived ATP production to 45 % (p = 0.0012) in WT and LdU^−/+^AB, but had little or no effect on LdU^−*/*+^ parasites. This result demonstrates that there is no probability of oxidative phosphorylation through succinate in the absence of LdUMSBP. Use of α-ketoglutarate and pyruvate in the reaction did not affect the ATP production in the absence of LdUMSBP and this data suggested that these molecules were not involved in substrate level phosphorylation (Fig. 7d). When we inhibit ATP production using all three different substrates by the attractyloside in the assay, the level of ATP production was at background level. These results indicate that LdUMSBP indirectly controls the oxidative phosphorylation pathway to generate ATP by controlling complex-III activity of ETC.

**Fig. 7:** Effect of UMSBP deletion on amastigote survival both in macrophages and in mice by interfering with electron transport chain, oxidative phosphorylation and ATP generation. **a** Image of isolated amastigotes from infected macrophages. **b** mRNA level of Cyt. b in WT, LdU^−*/*+^ and LdU^−/+^AB amastigotes by semiquantitative-RT-PCR. **c**  % of ATP production in mitochondria of WT, LdU^−*/*+^ and LdU^−/+^AB amastigotes. **d** ATP production by mitochondria from the indicated intracellular amastigotes was evaluated for three substrates (succinate, α-ketoglutarate and pyruvate, each indicating a separate mitochondrial pathway). The tested substrate is indicated at *top*. Addition of these compounds to the samples or no inhibitor (none) is indicated by the *bar graphs* *shading* according to the legend. ATP production in mitochondria of WT cells without addition of malonate or attractyloside was set to 100 % for each substrate. **e**–**f** Viability of amastigotes inside human macrophages after knocking out LdUMSBP as well as after complementation of WT UMSBP in LdU^−/+^ parasites (LdU^−/+^AB). **e** *Graph* showing the numbers of infected macrophages for the indicated parasites. **f** *Graph* showing the numbers of amastigotes in infected macrophages for the indicated parasites. **g** Survival of WT, LdU^−*/*+^ and LdU^−/+^AB parasites in BALB/c mice. Parasite burdens were analyzed at 6 or 14 weeks post-infection by serial dilution as described in “Methods” section. *Asterisk* denotes that the data are significant (p ≤ 0.001)

### LdU^−/+^ amastigotes are unable to survive in macrophages or mice

We found that LdUMSBP was important for mitochondrial oxidative phosphorylation through complex-III in amastigotes and therefore we wanted to explore whether this activity of LdUMSBP is important for leishmanial pathogenesis or not inside human macrophages and in BALB/c mice. Knockout of **s**ingle allele of LdUMSBP (LdU^−*/*+^) has no effect on the survival of promastigotes but, sufficient to diminish the growth of amastigotes inside macrophages (Fig. 7e, f, and Additional file 1: Figure S7). We then infected the macrophages with WT, LdU^−/+^ and LdU^−/+^AB promastigotes and the level of infection for all these cases were found to be similar at early hours of infection. With the progression of days, the burden of LdU^−/+^ amastigotes were decreasing gradually (p < 0.0001) inside the macrophages, while LdU^−/+^AB parasites replicated and survived as WT inside the host cells (Figs. 7e, f and Additional file 1: Figure S7). In LdU^−/+^ infected macrophages few viable amastigotes were found after 7 days of infection and that may be due to lower level of Complex-III activity in the absence of LdUMSBP. Therefore, LdUMSBP is essential for amastigotes survival inside macrophage and thereby indicating its post replication role [17].

In in vivo studies, we infected the BALB/c mice (n = 3) with 3 × 10^6^ metacyclic promastigotes of WT, LdU^−/+^ and LdU^−/+^AB parasites. After 6 and 14 weeks of infection, infected BALB/c mice were sacrificed and the parasite load was determined from both liver and spleen [31]. However, after 6 weeks of infection, LdU^−/+^ parasites survive at very lower rate and after 14 weeks, it did not survived inside the mice showing a significant (p < 0.0001) reduction of parasite burden in both liver and spleen compared to WT parasite (Fig. 7g). However, after episomal complementation of WT allele in LdU^−/+^ parasites (LdU^−/+^AB parasites), the survival rate of LdU^−/+^ parasite was reverted back to the WT level at 6 and 14 weeks in both liver and spleen (Fig. 7g). These results clearly conferred that LdUMSBP is essential for parasite survival and growth in the mammalian host.

## Discussion

UMSBP, a single-stranded DNA-binding protein recognises 12-nucleotide conserved sequence, UMS at the replication origin of kDNA minicircles and initiate kDNA replication [11, 12]. Sequence analysis revealed that DNA binding zinc finger domains are conserved in LdUMSBP as in other trypanosomes (Fig. 1). Fluorescence study showed that LdUMSBP is a mitochondrial protein (Additional file 1: Figure S3). Insilco modelling and docking studies showed that LdUMSBP could bind specifically with the UMS of kDNA minicircle and in vitro binding studies support these phenomena (Fig. 1 and Additional file 1: Figure S1). Therefore, LdUMSBP can interact with origin sequence (UMS) of minicircle in *L. donovani* (Fig. 2). Our study showed that the redox potential controls the binding of LdUMSBP to UMS (Additional file 1: Figure S2) as proposed in *C. fasciculata* where redox regulation of UMSBP was coupled UMSBP’s DNA-binding activity [14]. Moreover, mitochondrial redox regulating enzymes, TXN and TXNPx regulates the oxidation and reduction status of LdUMSBP and thereby its UMS binding activity (Fig. 3) [14].

In *T. brucei*, the over-expression of CBRL had a novel negative effect on kDNA level through oxidation/inactivation of UMSBP, but the growth defects of CBRL over-expression can be rescued by over-expressing TXN [16]. In *L. donovani*, UMSBP gets oxidised upon over-expression of LdCBRL in vivo, leading to loss of minicircles which is accompanied by the loss of kDNA (Fig. 4). Thus, the whole kDNA replication might be regulated by redox. Co-overexpression of TXN rescued the CB + cells from kDNA loss by reduction/activation of LdUMSBP (Fig. 4). These results suggest that in *L. donovani* the redox state of UMSBP and consequently its DNA binding activity are modulated enzymatically involving TXN, TXNPx and CBRL with their opposing effects.

The RNAi study in *Crithidia* spp. showed the post-replication functions of UMSBP [17]. In *L. donovani*, UMSBP’s post-replication functions were assessed for the first time by genetically manipulating this protein. LdUMSBP deleted cells displayed a decreased level of kDNA (Fig. 5) and this phenomenon was also reported by Milman et al. [17]. This possibly suggests that LdUMSBP deleted cells were defective in kDNA replication. Mitochondrion harnesses its energy through the ETC complexes which passes the electrons to oxygen to carry out respiration which is essential for survival of both promastigotes and amastigotes of *Leishmania* [46]. The proton gradient produced by electron transport drives the F1/F0 ATPase to generate ATP by oxidative phosphorylation. Loss of kDNA in response to the deletion of UMSBP causes reduction in the activities of ETC complex-III [19] in *L. donovani*. In LdU^−/−^ parasites, loss of kDNA is linked with loss of activity of complex-III through the loss of Cyt.b (indispensible part of complex-III activity and encoded by kDNA). As the complex-III is involved in ATP synthesis, the level of intracellular ATP was decreased in LdU^−/−^ parasites and finally the rate of parasite viability was decreased (Fig. 5g). Both intracellular ATP production and parasite viability were restored near to WT after episomal expression of LdUMSBP in LdU^−/−^ parasites, specifically indicating the role of LdUMSBP in ATP production and parasite survival (Figs. 5g, 6c).

Normally, ETC-complexes function as proton pumps to maintain ∆Ψ_m_ [20]. Due to inactivation of complex-III in LdU^−/−^ parasites, ∆Ψ_m_ was decreased and consequently, the level of ATP was decreased (Fig. 6c, h). The change in ∆Ψ_m_ was accompanied by the release of Cyt.c from mitochondria to cytosol in LdU^−/−^ parasites (Fig. 6i) which causes apoptotic like phenomena [39]. Bifurcation of electrons from the mitochondrial complexes and interference in electron flow increase the intracellular ROS [47]. Moreover, inhibition of complex-III by antimycin-A induces ROS in *L. donovani* [20]. Similarly, in LdU^−/−^ parasites, complex-III activity was disrupted due to loss of Cyt.b and consequently, electron flow was hindered and therefore, the level of ROS was increased (Fig. 6g) which induces apoptotic like death in LdU^−/−^ parasites, as demonstrated by PS externalization, metacaspase like protease activity and DNA fragmentation (Fig. 6d–f, j) [20, 33]. Intracellular level of ROS, ∆Ψ_m_, Cyt. b, PS externalization and DNA fragmentation were restored back to the WT level after episomal expression of LdUMSBP in LdU^−/−^ which specifically implicates that UMSBP of *L. donovani* has the role in parasite survival other than kDNA replication by regulating the apoptotic like phenomena by controlling the ETC and ATP production through Cyt.b.

Dyskinetoplastic *T. brucei* are incapable of completing their usual developmental cycle in the insect vector, due to their inability to perform oxidative phosphorylation. Nevertheless, they are usually virulent for their mammalian hosts as parasites with intact kDNA [48]. So, the role of LdUMSBP was studied in intracellular amastigotes. Functional LdUMSBP in amastigotes, correlated with complex-III activity is essential for *Leishmania* survival inside the human macrophages. Increased mitochondrial activity has the crucial role in the survival of amastigotes inside host cells [49, 50]. For production of energy, intracellular amastigotes are more dependent on the tricarboxylic acid cycle and mitochondrial respiration than on glycolysis [51]. Our study demonstrated that LdU^−*/*+^ parasites do not proliferate in human macrophages and in mouse (Fig. 7). This phenomenon in LdU^−/+^ parasites is due to inactivation of complex-III (Table 1) due to loss of Cyt.b, along with reduced ATP production by oxidative phosphorylation (Fig. 7). Both replication in macrophages and virulence in mice were restored as in WT by episomal expression of WT LdUMSBP in LdU^−*/*+^ parasites (LdU^−/+^AB) and these results clearly demonstrating LdUMSBP as a virulence factor for amastigotes.

From the data, it can be summarized that in *Leishmania* the kDNA binding activity of LdUMSBP is regulated by mitochondrial multi enzymes system. Other than kDNA replication initiation, we have shown probably for the first time that LdUMSBP is involved in apoptosis by controlling the ETC and ATP synthesis through Cyt.b and consequently regulates amastigotes survival inside human macrophages and virulence in mice by controlling ETC and oxidative phosphorylation (Fig. 8).

**Fig. 8:** Model representing the functional regulation of LdUMSBP during kDNA replication and its role in electron transport chain, apoptosis, oxidative phosphorylation and amastigotes survival. The trypanothione upon reduction by trypanothione reductase (TR) reduces tryparedoxin (TXN). Reduced TXN reduces UMSBP, tryparedoxin peroxidise (TXNPx) and CBRL. Reduced LdUMSBP binds with UMS of minicircle and kDNA replication initiates, whereas its oxidation impairs the binding with UMS. The CBRL, TXN and TXNPx regulate the binding activity of LdUMSBP with their opposite effects. Over expression (OE) of CBRL induces oxidation of UMSBP which results kDNA loss. Co-overexpression of TXN rescues the parasites from this negative effect. UMSBP knockout in *L. donovani* leads to kDNA loss which in turn reduces the level of Cyt. b and complex-III of Electron Transport Chain is inhibited and consequently ATP generation (oxidative phosphorylation) is impaired and parasite survival is reduced through apoptosis in response to complex-III inhibition. Also, the impairment of oxidative phosphorylation and ATP generation reduces the amastigotes survival as well as its virulence in BALB/c mice. *UMSBP* *ox* oxidized UMSBP, *UMSBP* *red* reduced UMSBP, *TXN(S)*_*2*_ oxidized TXN, *TXN(SH)*_*2*_ reduced TXN

The functional characterization of a protein specifically important for kDNA replication in *Leishmania*, required for survival and intracellular proliferation of amastigotes in the mammalian host is an important step towards understanding this human pathogen and developing means to control it. Drugs aimed at disrupting the function of LdUMSBP which has no orthologue in the human cell, may be a way for clearing the parasites. It is reported that mutations in Cyt. b gene of ETC alters the sensitivity of MDR1 and regulates resistance level to anti-parasitic drugs [52]. As the LdUMSBP regulates the amastigotes survival by controlling ETC activity and oxidative phosphorylation through the expression level of Cyt.b, it may regulates indirectly the activity of MDR1 and thereby may regulates the reported MDR1 mediated AmB resistance property [33]. Our lab is now working in this direction to investigate the role of LdUMSBP in AmB resistance property. Moreover, kDNA replication machinery has the ability to be used as a potential drug targets in *Trypanosoma* [53]. Therefore, LdUMSBP can be used as a future chemotherapeutic option for VL. In addition, the LdU^−/+^ cell line, which proliferates well as promastigotes and shows little or no pathogenesis in mice could be further investigated as a possible genetically modified live attenuated *Leishmania* vaccine. Through our initial study we have seen that the vaccination with a single i.p. injection of LdU^−/+^ single knockout parasites elicits complete protection against WT parasite challenge (unpublished data). Studies are underway to evaluate protective immunity conferred by LdU^−/+^ single gene-deleted parasites in animal models against challenge by virulent *Leishmania* parasites.

## Conclusion

From the results it can be concluded that the kDNA binding activity of UMSBP is regulated by cellular redox signalling mechanism. For the first known time we have shown that deletion of UMSBP induces kDNA loss which causes apoptosis like death through interfering with Electron Transport Chain and regulates the virulence of *L. donovani* in macrophages and mice by disrupting Oxidative Phosphorylation. The increasing trend of resistance towards the current chemotherapy for Visceral Leishmaniasis (VL), suggests the urgent need of a novel and potential molecule which can be exploited as drug target. To achieve this goal, UMSBP can be considered as valuable and potential target because of its uniqueness compared to the host and also required for survival and intracellular proliferation of amastigotes in the mammalian host.

## Additional file

10.1186/s13578-016-0072-z 3D Model of LdUMSBP designed by Bio-informatics tools. **Figure S2.** Expression, Purification of recombinant LdUMSBP and Generation of anti-LdUMSBP Antibody. **Figure S3.** Immunolocalization of LdUMSBP in kDNA disk demonstrated by Phase and Fluorescence Microscopy. **Figure S4.** Redox potential controls oxidation-reduction status of UMSBP and its binding activity. **Figure S5.** PCR amplification of HYG and NEO gene from LdU^−/−^ parasites, confirming the successful deletion of two allele of UMSBP by the Hygromycin and Neomycin cassette. **Figure S6.** Southern blot to demonstrate the deletion of two alleles of LdUMSBP from L. donovani genome. **Figure S7.** Phase contrast microphotograph after Geimsa staining of infected macrophages [infected with wild type (R), single knock out LdUMSBP (LdU^−/+^) and double knock out LdUMSBP (LdU^−/−^). **Table S1.** List of Primers. **Table S2.** Interacting amino acids of LdUMSBP with UMS sequence in docking study.
